# GNAO1 as a Novel Predictive Biomarker for Late Relapse in Hepatocellular Carcinoma

**DOI:** 10.1155/2021/7631815

**Published:** 2021-11-30

**Authors:** Meiling Du, Jie Feng, Yiran Tao, Qincong Pan, Fengyuan Chen

**Affiliations:** ^1^Department of Gastroenterology, Shanghai Fifth People's Hospital, Shanghai 201200, China; ^2^Department of General Medicine, Zhoupu Community Health Service Center, Shanghai 201100, China

## Abstract

GNAO1, the alpha O1 subunit of *G* protein, was reported to be significantly downregulated in hepatocellular carcinoma (HCC), as well as being implicated in a variety of intracellular biological events; findings suggest that it may act as a tumor suppressor. Our goal was to further explore the expression of GNAO1 in HCC patients and its potential clinical significance. Oncomine and Kaplan–Meier plotter databases were used to assess the mRNA expression of GNAO1 in HCC tissues and patient survival time. Subsequently, immunohistochemistry (IHC) was used to measure GNAO1 protein level in tissue from 79 cases of HCC and paired adjacent tissues. The Kaplan–Meier survival analysis, Cox regression model, and prognostic nomogram were used to evaluate the prognostic role of GNAO1 in HCC. Results demonstrated that mRNA and protein expressions of GNAO1 were both lower in HCC tissues than in adjacent tissues (all *p* < 0.01). HCC patients with high expression of GNAO1 had better relapse-free survival (RFS) than those with low GNAO1 expression (all *p* < 0.05). A high expression of GNAO1, meanwhile, functioned as a good predictor of late relapse for HCC (*p* < 0.05). The nomogram consisting of GNAO1 expression and the tumor-node-metastasis (TNM) model presented good ability in predicting the 3-year relapse for HCC (C-index = 0.614). In conclusion, GNAO1 was a reliable biomarker of relapse prediction for HCC.

## 1. Introduction

Liver cancer is one of the most lethal and prevalent cancers worldwide and has recently become the third leading cause of cancer-related mortality in humans [1]. Hepatocellular carcinoma (HCC) is the primary cancer of the liver, accounting for almost 75% of all liver cancers globally [2]. Established major risk factors for HCC include chronic infection with hepatitis B virus (HBV) and hepatitis C virus, excess alcohol consumption, and nonalcoholic fatty liver disease. Despite of recent progress in diagnosis and treatment, the clinical outcomes of HCC patients remain very poor. Thus, it is particularly crucial to explore a novel biomarker of early diagnosis or prognostication for HCC.

GNAO1 encodes the alpha O1 subunit of guanine nucleotide-binding proteins, which can trigger signaling cascades and regulate several cellular events when they bind to a serpentine receptor [3]. GNAO1, first mentioned in 1987 [4], is located on chromosome 16q13 and is predominantly localized in nervous tissues and neuroendocrine cells [5]. Previous research focused on GNAO1 mutation-induced encephalopathy, including hypotonia, epilepsy, and dyskinesia [6–9]. Additionally, GNAO1 dysfunction or aberrant expression could promote oncogenesis such as in gastric cancer [10], colorectal cancer [11, 12], and breast cancer [13].

As an association with HCC, Pei et al. found that GNAO1 was downregulated in HCC cells and that the silencing of GNAO1 by small-interfering RNA increased the proliferation, while inhibiting the senescence of HCC cells [14]. Lately, researchers, including our own team, further elucidated that low expression of GNAO1 in HCC cells was partly attributed to DNA methyltransferase 1 and the deacetylase silent information regulator 1 indirectly mediating the promoter hypermethylation [15, 16]. In clinical study, Pei et al. also demonstrated that GNAO1 was comparably less in HCC tissues than in adjacent tissues by immunohistochemistry (IHC) on 20 paired samples [14]. However, very small sample size and absence of a statistical test in the study are incomplete for us to understand the expression of GNAO1 in HCC patients. Moreover, the potential clinical significance of GNAO1 remains unknown.

In our study, bioinformatics data were studied, with the IHC assay aiming to define the trait and the role of GNAO1 in HCC patients, based on the effective statistical analysis. We hope to provide a good prognostic biomarker and a new target for anticancer therapy in HCC.

## 2. Materials and Methods

### 2.1. Oncomine Database Analysis

The differential expression of GNAO1 mRNA between HCC and normal liver tissues was reviewed in the Oncomine database (https://www.oncomine.org/resource/login.html), which is a cancer microarray database and web-based data-mining platform aimed at facilitating discovery from genome-wide expression analysis [17]. The threshold settings were as follows: gene ranking of top 10%, a fold change of 2.0, and a *p* value of 1E-4.

### 2.2. Kaplan–Meier Plotter Database Analysis

The Kaplan–Meier plotter database (http://www.kmplot.com), an online survival analysis tool, was used to evaluate relationships between gene expression and patient prognosis, such as overall survival (OS) and relapse-free survival (RFS), across a large collection of publicly available cancer microarray datasets [18]. Patient samples were split into two groups according to the best cutoff of GNAO1 expression (low versus high expression) and were assessed by a Kaplan–Meier survival plot, with the hazard ratio (HR) with 95% confidence interval (CI) and log rank *p* value.

### 2.3. Clinical Samples

A human liver cancer tissue microarray (cat no. LVC1605) containing paired tumor and normal tissue from 80 cases, together with patient clinical data, was purchased from Shanghai zhuolibiotech Co., Ltd. (Shanghai, China). All patients received radical surgery from January 2004 to June 2012. Patients who were pathologically diagnosed with primary HCC were adopted into the study. Exclusion criteria were a history of radiotherapy or chemotherapy before surgery and less than 36 months of follow-up.

### 2.4. IHC Assay

According to the instructions of the UltraSensitive SP detection kit (KIT-9730, Maxim Biotech, Fuzhou, China), IHC staining was performed on HCC tissue microarray to detect the expression of GNAO1 protein. Briefly, tissue sections were deparaffinized with xylene and rehydrated, followed by microwave antigen retrieval. After being blocked with hydrogen peroxidase and nonimmune animal serum, the sections were incubated at 4°C overnight with the primary antibody against GANO1 (1 : 200, #12635-1-AP, Proteintect Group, Rosemont, USA). The sections were further incubated in the solution of biotin-labeled secondary antibody at room temperature for 30 minutes and then in streptavidin peroxidase reagent for 10 minutes. The sections should be rinsed in PBS thrice after each step (each rinse for five minutes). Finally, IHC staining was conducted using a DAB kit (P0203, Beyotime Biotech, Shanghai, China).

### 2.5. Semiquantitative Analysis

The immunohistochemical staining result was evaluated using a semiquantitative method (immunoreactive score, IRS) as described previously [19]. IRS (0–12) for each slice was calculated by multiplying the staining intensity in four gradations (0, negative; 1, weak; 2, moderate; and 3, strong) with the percentage of positive cells in five gradations (0, negative; 1, ≤ 10%; 2, 11–50%; 3, 51–80%; and 4, ≥81%), and each specimen was measured in three different magnification fields. Two pathologists independently observed the staining results under double-blind conditions.

### 2.6. Statistical Analysis

Statistical analysis was made in SPSS (version 22.0) software and *R* (version 4.1.0.) software. The measurement data with normal distribution were expressed as means ± standard deviations, and nonnormally distributed data were expressed as the median. We performed Student's *t*-test and Pearson's chi-squared test to compare the difference between groups. Moreover, Kaplan–Meier curves were drawn to compare the prognostic difference between groups. The prognostic performance of factors was explored via univariable and multivariable Cox proportional hazard regression analysis. Then, the predictive performance of factors was assessed via time-dependent receiver operating characteristic (ROC) curves and the area under the curve (AUC) by using the “survival ROC” package of *R* software. Nomogram, a powerful tool for quantifying each prognostic factor on the survival [20], was created based on the Cox regression model by using the “rms” package. The calibration curve and C-index were generated to analyze the agreement between the nomogram and ideal observation. *p* value less than 0.05 was considered statistically significant.

## 3. Results

### 3.1. Patient Characteristics

A total of 79 cases of primary HCC were adopted into the group, with the median follow-up of 42 months (range: 5–84 months). The median age of patients at diagnosis was 54 years, and 17 (21.5%) patients were aged 60 years and older. Sixty-six patients (83.5%) were male, and 13 (16.5%) were female. The number of patients with tumor stage I, II, III, and IV was 30 (38.0%), 34 (43.0%), 3 (3.8%), and 12 (15.2%), respectively. Detailed clinical parameters of 79 HCC patients are shown in Table 1.

### 3.2. Low mRNA and Protein Levels of GNAO1 in HCC Tissues

There were 5 RNA chips with a total of 413 HCC and 340 normal liver tissues involved in the analysis of differential expression of GNAO1 mRNA in the Oncomine database. Results showed that the mRNA expression of GNAO1 was significantly lower in HCC tissues than in normal liver tissues (Figure 1).

To confirm the predictive results, IHC assay on 79 paired HCC samples was performed to examine GNAO1 protein level. The mean ± standard deviation IRS of GNAO1 in cancerous tissues and noncancerous tissues was 6.43 ± 3.93 and 10.95 ± 2.25, respectively. The IRS of GNAO1 in the tumor was much lower than that in adjacent tissues (*t* = 9.840, *p* < 0.001; Figure 2), indicating that the protein expression of GNAO1 was significantly lower in HCC tissues than in adjacent tissues. Results also showed that GNAO1 protein was mainly distributed on the membrane and in the cytoplasm of liver cells.

### 3.3. Relationships between GNAO1 Expression and Patient Clinicopathological Parameters

In our study, the median IRS scores of GNAO1 in 79 HCC tissues was 8. IRS ranged from 0 to 12, with IRS ≥8 indicating high GNAO1 expression and IRS <8 indicating low GNAO1 expression. There were 44 patients with high expression of GNAO1 and 35 patients with low expression of GNAO1. As shown in Table 1, the differential expression of GNAO1 protein (low versus high) was not significantly associated with patient clinical characteristics, including age, sex, HBV infection, alpha-fetoprotein values, and liver cirrhosis, as well as pathological data, including tumor location, tumor size, tumor number, tumor type, vascular invasion, and tumor-node-metastasis (TNM) stage.

### 3.4. High GNAO1 Expression Was Associated with Favorable RFS in HCC

In the Kaplan–Meier plotter database, the RFS analysis of all HCC patients (*n* = 316), stage I-II (*n* = 228), and stage III-IV (*n* = 70) revealed that patients with high mRNA expression of GNAO1 had more favorable RFS than those with low GNAO1 expression (all *p* < 0.05; Figures 3(a)–3(c)).

We also analyzed the IHC staining results and found that RFS of HCC patients with high expression of GNAO1 protein was significantly better than those with low GNAO1 expression (all *p* < 0.05; Figures 3(d)–3(e)). The average RFS in the high GNAO1 expression cohort was longer than that in the low GNAO1 expression cohort (31.36 ± 22.97 vs. 20.31 ± 13.38 months, *p* < 0.01).

### 3.5. GNAO1 Was a Reliable Biomarker for Relapse Prediction in HCC

Both univariate and multivariate Cox regression analysis indicated that GNAO1 expression was a negative factor significantly associated with HCC relapse (HR = 0.512, 95% CI = 0.297–0.882, *p* < 0.05; HR = 0.420, 95% CI = 0.237–0.744, *p* < 0.01, respectively; Table 2). Subsequently, ROC analysis was conducted to assess how GNAO1 expression could behave in predicting relapse. As shown in Figure 4(a), the AUC of GNAO1 expression performed on relapse was 0.688, which was superior to that of TNM stage (0.606) and other clinicopathological parameters.

To predict the probability of 1-, 2-, and 3-year relapse, a nomogram model was established (Figure 4(b)). Calculating the score of GNAO1 expression and TNM stage, a straight line was generated to evaluate the relapse probability at each time point. The calibration curve presented that the rate of predicted relapse in 3-year closely paralleled the actually observed ratio (C-index = 0.614; Figure 4(c)), indicating the agreement between model prediction and reality.

## 4. Discussion

Most information about GNAO1 in HCC stems from in vitro experiments and is, as yet, insufficient to really understand the function of GNAO1. In our study, we analyzed GNAO1 expression and its clinical significance in HCC patients by using bioinformatics data, IHC assay, and effective statistical analysis.

A total of 5 RNA chip analysis, involving 413 HCC and 340 normal liver samples, all revealed that GNAO1 mRNA expression was at a lower level in HCC tissues than in normal liver tissues. Meanwhile, GNAO1 protein expression was confirmed to be significantly downregulated in HCC tissues by IHC on 79 paired samples, concurring with the bioinformatics results and the report of Pei et al. [14].

Subsequently, a survival analysis was conducted using data from the Kaplan–Meier plotter database along with IHC results. The analysis showed that HCC patients with high GNAO1 expression had better RFS compared to those with low GNAO1 expression, regardless of whether the tumor was at an early or advanced stage. This result may be attributed to the biological function of GNAO1 in HCC cells, which inhibits proliferation and promotes apoptosis and senescence [14–16]. Notably, the range of RFS from IHC results was shorter than that in the database, which may be related to the short postoperative follow-up time of our patients. Besides, it is interesting that HCC patients with high GNAO1 expression did not have prolonged OS (Figure 5). It is well known that OS is not only affected by tumor relapse but is also subject to other factors, such as how the patient responds to retreatment [21].

In general, TNM stage is a systematic anatomic-based classification that provides a method to estimate cancer prognosis. It is believed that early-stage patients have better outcomes after surgical resection [22, 23]. In our study, TNM stage was not closely related to GNAO1 expression. However, the Cox regression model and ROC analysis demonstrated that early TNM stage and high GNAO1 expression were two independent predictors of late relapse in HCC patients, with GNAO1 expression predicting relapse more accurately. Besides, the AUC of TNM stage performed on HCC relapse was 0.606 in our study, which was similar to the result (0.616) reported by Liu et al. [24]. Furthermore, we successfully constructed a valuable prognostic model by combining GNAO1 expression with TNM stage to more precisely predict the likelihood of relapse in HCC patients. The results demonstrated that the GNAO1 related prognostic model can be used to predict HCC relapse within 3 years, and patients with high GNAO1 expression and early tumor stage have a low relapse rate. Bu et al. constructed a similar prognostic model to predict survival of patients after colorectal cancer surgery, which has great potential to be used in the real world [25].

There were several limitations in the study. We did not analyze the RFS of 15 patients with advanced HCC in the IHC assay. However, it can be concluded from the analysis of the Kaplan–Meier plotter database that advanced patients with high GNAO1 expression also have better RFS. Besides, our HCC tissues were mainly obtained from patients suffering from the HBV (62/79), which is the leading cause of HCC in China [26], and the GNAO1 prognostic model was constructed based on retrospective data. Hence, a rich supply of different HCC samples with long-term follow-up information are required to further study the clinical significance of GNAO1, including verifying its prognostic value by recruiting a prospective cohort.

## 5. Conclusions

Our findings provide convincing evidence that GNAO1 is significantly downregulated in HCC tissues and GNAO1 expression can satisfactorily predict HCC relapse. Furthermore, the nomogram consisting of GNAO1 expression and the TNM model presents good ability in predicting the 3-year relapse, suggesting that it could be a reliable biomarker of relapse prediction as well as a promising therapeutic target for HCC.

## Figures and Tables

**Figure 1:** Expression of GNAO1 mRNA was lower in HCC tissues than in normal liver tissues based on the Oncomine data. Research samples were Wurmbach Liver (*t* = 10.249, *p*=4.069*E* − 13), Roessler Liver 2 (*t* = 21.263, *p*=1.440*E* − 66), Roessler Liver (*t* = 5.363, *p*=6.000*E* − 6), Chen Liver (*t* = 3.164, *p*=0.002), and Mas Liver (*t* = 3.409, *p*=0.002), respectively. ^*∗∗∗*^*p* < 0.001, ^*∗∗*^*p* < 0.01.

**Figure 2:** Expression of GNAO1 protein was lower in HCC tissues than in adjacent normal tissues based on the IHC results. (a) Representative high expression of GNAO1 in adjacent tissue, magnification: ×400; (b) representative low expression of GNAO1 in HCC tissue, magnification: ×400; and (c) the IRS in HCC tissues was statistically lower than that in adjacent normal tissues (*t* = 9.840, *p*=2.567*E* − 15). ^*∗∗∗*^*p* < 0.001.

**Figure 3:** The Kaplan–Meier curves of RFS of HCC patients based on GNAO1 expression (low versus high). (a–c) RFS analysis of all HCC patients (*n* = 316), stages I-II (*n* = 228), and stages III-IV (*n* = 70) in the Kaplan–Meier plotter database; (d–e) RFS analysis of all HCC patients (*n* = 79) and stages I-II (*n* = 64) based on the IHC results.

**Figure 4:** Construction of a prognostic model for HCC relapse assessment. (a) ROC analysis for GNAO1 expression and clinicopathologic parameters; (b) prognostic nomogram for HCC patients; and (c) calibration curves for the nomogram at 3 years.

**Figure 5:** Kaplan–Meier curves of OS of HCC patients based on GNAO1 expression (low versus high). (a–c) OS analysis of all HCC patients (*n* = 364), stage I-II (*n* = 253), and stage III-IV (*n* = 87) in the Kaplan–Meier plotter database; (d–e) OS analysis of all HCC patients (*n* = 79) and stage I-II (*n* = 64) based on the IHC results.

**Table 1:** Relationships between GNAO1 protein level and clinicopathological parameters in 79 HCC patients.

Clinicopathological parameters	Case, *n* (%)	GNAO1 expression		*p* value
		Low (*n* = 35)	High (*n* = 44)	
Age (years)				
<60	62 (78.5)	29	33	0.399
≥60	17 (21.5)	6	11	

Sex				
Male	66 (83.5)	29	37	0.883
Female	13 (16.5)	6	7	

HBV infection				
Yes	62 (78.5)	26	36	0.418
No	17 (21.5)	9	8	

AFP				
<200 ng/mL	30 (38.0)	16	14	0.206
≥200 ng/mL	49 (62.0)	19	30	

Liver cirrhosis				
Yes	55 (69.6)	26	29	0.421
No	24 (30.4)	9	15	

Tumor location				
Left lobe	42 (53.2)	16	26	0.237
Right lobe	37 (46.8)	19	18	

Maximum tumor size				
<30 mm	13 (16.5)	8	5	0.171
≥30 mm	66 (83.5)	27	39	

Number of tumors				
1	72 (91.1)	32	40	0.751
≥2	7 (8.9)	3	4	

Tumor type				
Lump	71 (89.9)	30	41	0.473
Nodular	8 (10.1)	5	3	

Vascular invasion				
Yes	26 (32.9)	11	15	0.802
No	53 (67.1)	24	29	

TNM stage (AJCC 8th)				
I-II	64 (81.0)	31	33	0.215
III-IV	15 (19.0)	4	11	

Abbreviations: HCC: hepatocellular carcinoma, HBV: hepatitis B virus, AFP: alpha-fetoprotein, TNM: tumor-node-metastasis, AJCC: American Joint Committee on Cancer

**Table 2:** Cox survival analysis of GNAO1 protein level and clinicopathological parameters in 79 HCC patients

Parameters	Univariate		Multivariate	
	HR (95% CI)	*p* value	HR (95% CI)	*p* value
GNAO1 level (low vs. high)	0.512 (0.297–0.882)	**0.016** ^*∗*^	0.420 (0.237–0.744)	**0.003** ^*∗∗*^
Age (years) (<60 vs. ≥60)	0.947 (0.498–1.800)	0.868		
Sex (male vs. female)	1.442 (0.680–3.057)	0.340		
HBV infection (yes vs. no)	0.821 (0.445–1.514)	0.527		
AFP (ng/mL) (<200 vs. ≥200)	0.672 (0.392–1.153)	0.149		
Liver cirrhosis (yes vs. no)	0.841 (0.474–1.492)	0.553		
Tumor location (left vs. right)	1.101 (0.644–1.881)	0.725		
Maximum tumor size (mm) (<30 vs. ≥30)	1.156 (0.545–2.452)	0.706		
Number of tumors (1 vs. ≥2)	0.853 (0.340–2.144)	0.736		
Tumor type (lump vs. nodular)	0.590 (0.213–1.683)	0.311		
Vascular invasion (yes vs. no)	1.245 (0.718–2.157)	0.436		
TNM stage (I-II vs. III-VI)	1.959 (1.055–3.638)	**0.033** ^*∗*^	2.581 (1.345–4.954)	**0.004** ^*∗∗*^

Abbreviations: HCC: hepatocellular carcinoma, HR: hazard ratio, CI: confidence interval, HBV: hepatitis B virus, AFP: alpha-fetoprotein, TNM: tumor-node-metastasis. ^*∗∗*^*P* < 0.01, ^*∗*^*P* < 0.05.

## Data Availability

The datasets used in this paper are available from the corresponding author upon request.
